# Non-thermal plasma inhibits human cervical cancer HeLa cells invasiveness by suppressing the MAPK pathway and decreasing matrix metalloproteinase-9 expression

This article has been retracted.

**DOI:** 10.1038/srep19720

**Published:** 2016-01-28

**Authors:** Wei Li, K. N. Yu, Lingzhi Bao, Jie Shen, Cheng Cheng, Wei Han

**Affiliations:** 1 Center of Medical Physics and Technology, Hefei Institutes of Physical Sciences, Chinese Academy of Sciences, 350 Shushanhu Road, Hefei, 230031, Anhui Province, P.R. China.; 2 Institute of Plasma Physics, Hefei Institutes of Physical Sciences, Chinese Academy of Sciences, 350 Shushanhu Road, Hefei, 230031, Anhui Province, P.R. China.; 3 Department of Physics and Materials Science, City University of Hong Kong, Tat Chee Avenue, Kowloon Tong, Hong Kong; 4 Collaborative Innovation Center of Radiation Medicine of Jiangsu Higher Education Institutions and School for Radiological and Interdisciplinary Sciences (RAD-X), Soochow University, Suzhou, Jiangsu, China

## Abstract

Non-thermal plasma (NTP) has been proposed as a novel therapeutic method for anticancer treatment. However, the mechanism underlying its biological effects remains unclear. In this study, we investigated the inhibitory effect of NTP on the invasion of HeLa cells, and explored the possible mechanism. Our results showed that NTP exposure for 20 or 40 s significantly suppressed the migration and invasion of HeLa cells on the basis of matrigel invasion assay and wound healing assay, respectively. Moreover, NTP reduced the activity and protein expression of the matrix metalloproteinase (MMP)-9 enzyme. Western blot analysis indicated that NTP exposure effectively decreased phosphorylation level of both ERK1/2 and JNK, but not p38 MAPK. Furthermore, treatment with MAPK signal pathway inhibitors or NTP all exhibited significant depression of HeLa cells migration and MMP-9 expression. The result showed that NTP synergistically suppressed migration and MMP-9 expression in the presence of ERK1/2 inhibitor and JNK inhibitor, but not p38 MAPK inhibitor. Taken together, these findings suggested that NTP exposure inhibited the migration and invasion of HeLa cells *via* down-regulating MMP-9 expression in ERK1/2 and JNK signaling pathways dependent manner. These findings provide hints to the potential clinical research and therapy of NTP on cervical cancer metastasis.

Non-thermal plasma (NTP), generated at room temperature by ionization of neutral gas molecules, results in a mixture of numerous short-lived but highly active chemical species^1^. These active chemical species are essential for various biological processes in cells and human tissues. In recent years, NTP have been used in many biomedical applications such as wound healing, sterilization, blood coagulation and the ablation of cultured liver cancer cells^2^,^3^,^4^,^5^. In addition, newly developed NTP exert anti-tumor effects in various cancer cell types both *in vitro* and *in vivo*^6^,^7^,^8^,^9^. These researches present exciting prospects for potential clinical applications of NPT on cancer therapy. Many studies have shown that NTP treatment induce apoptosis in various tumor models^6^,^10^,^11^. Further studies also demonstrate that NTP treatment inhibits colorectal and thyroid papillary cancer cells invasion and metastasis *in vitro*^12^,^13^,^14^. However, the underlying molecular signaling pathways for NTP-inhibited migration and invasion in cancer cells still need further investigation.

Cervical cancer is the second leading cause of cancer-related mortality in women worldwide, accounting for approximately 270,000 deaths per year^15^,^16^. Approximately 50% of cervical cancer patients die from metastasis after treatment with the current main therapeutic methods^15^. Cancer metastasis, spreading of cancer cells from the primary neoplasm to distant sites, forms the secondary tumor^17^. Metastasis occurs *via* a complex series of events, including invasion of cells from a primary tumor into the circulation system, immigration of these cells to distant organs, adhesion to endothelial cells, and infiltration into tissue^17^,^18^. In this process, degradation of the extracellular matrix (ECM) is mainly performed by matrix metalloproteinases (MMPs)^19^. In the MMP family, MMP-2 and MMP-9 are crucial for the invasion and metastasis of many types of cancer cells, and so several inhibitors of MMPs have been tested in clinical trials for prevention of tumor invasion and metastasis^20^,^21^,^22^. The expression and activity of MMP-9 and MMP-2 are regulated by various growth factors or mitogen-activated protein kinase (MAPK)^23^,^24^. Many studies have demonstrated that MAPKs, including extracellular signal-regulated kinase (ERK1/2), c-Jun N-terminal kinase (JNK), and p38 MAPK, play important regulatory roles in cell invasion and metastasis^24^. As such, inhibition of MAPKs pathway is considered potential targets for preventing cancer metastasis.

In this study, we explored the inhibitory effects and the possible underlying molecular mechanisms of NTP on the migration and invasion of human cervical cancer HeLa cells. Our results demonstrated that NTP exposure inhibited the migration and invasion of human cervical cancer HeLa cells *via* inhibiting MAPK signaling pathway, which led to down-regulation of MMP-9 activity and expression. These findings provided a novel mechanistic insight into the potential of NTP on the suppression of cervical cancer invasion and metastasis.

## Results

### NTP inhibited proliferation of HeLa cells

In this study, a non-thermal plasma (NTP) generating system was developed in our lab as previously described^25^. Helium gas was injected into the chamber through the gas inlet with a fixed flow rate of 80 L/h. In order to expel as much air as possible from the reactor chamber, helium was injected at 5 min before the experiment. The non-thermal plasma was generated by a voltage of 12 kV (peak to peak) at a frequency of 24 kHz.

Previous reports showed that NTP induced cell death in a exposure time dependent manner^26^. To determine the effect of NTP exposure time on the viability of Hela cells, the CCK-8 assay was used to measure cell viability. A gas-only treatment (helium) was used as a reference to exclude the gas effects of NTP. The results of the CCK-8 assay are shown in Fig. 1. The results showed that after 24 or 48 h incubation, NTP exposure from 10 to 40 s induced no distinct cytotoxic effects on HeLa cells (*p* > 0.05; Fig. 1). With the increase of exposure time (60 or 80 s), the cell viability decreased when compared with the control group (i.e., cells without NTP treatment) (*p* < 0.05; Fig. 1). However, for longer-time incubation (72 h), NPT exposures for 40 s significantly decreased the cell viability when compared with the control group (*p* < 0.05; Fig. 1). Therefore, NTP exposure durations of 10, 20 or 40 s were used in the subsequent experiments.

In addition, after 24 h incubation, NTP exposures from 10 to 40 s did not affect DNA damages (Fig. 2a). Flow cytometry analysis of apoptosis and mitochondrial transmembrane potential (Δψm) showed that NTP exposures from 10 to 40 s had no significantly effects on cell apoptosis and mitochondrial transmembrane potential (*p* > 0.05; Fig. 2b,c). Cytoskeleton staining also showed that NTP exposures from 10 to 40 s did not change cellular morphology or cytoskeletal architecture (Fig. 2d). Western blot analysis showed that NTP treatment had no effects on the expressions of Bax, Bcl-2, Caspase-3, Bid, cytochrome *c* and γ-H2AX (Fig. 3). Taken together, after 24 h incubation, NTP exposure durations of 10, 20 or 40 s did not affect the viability of HeLa cells or cause physical damages to the cells.

### NTP inhibited migration and invasion of HeLa cells

The capabilities of migration and invasion of tumor cells are important characteristics of metastasis^18^. We first performed the wound-healing assay to measure the effect of NTP on HeLa cell motility. As shown in Fig. 4, NPT exposures significantly decreased the cell motility in a dose-dependent manner. NPT exposures for 20 or 40 s inhibited cell migration by 63% or 45%, respectively, when compared with the control group.

Transwell migration assay and Matrigel invasion assay were also used to examine the effects of NTP on migratory and invasive capacities of HeLa cells. As shown in Fig. 4, NPT exposures significantly inhibited the migration of HeLa cells in an exposure time-dependent manner. The percentage of transwell migrated cells decreased to 54% or 31% with NTP exposures of 20 or 40 s, respectively (see Fig. 5). Similarly, NPT exposures significantly decreased the number of invading cells through the matrigel when compared with control group. NTP exposures for 20 or 40 s inhibited the number of cells from invading to the lower chamber by 34% or 23%, respectively. Taken together, these results suggested that NTP could inhibit the migration and invasion of HeLa cells.

### NTP decreased proteolytic activity and expression of MMP-9 in HeLa cells

Previous studies demonstrated that the expressions of MMP-2 and -9 were high in various malignant tumors and were closely related with tumor migration^27^,^28^. Therefore, in order to further test whether NTP treatment suppressed HeLa cell invasion *via* affecting the expression of matrix metalloproteinase, gelatin zymography assay was performed to measure MMP-9 and MMP-2 activities. As shown in Fig. 6a, NTP treatment significantly inhibited gelatinolytic activity of MMP-9 in an exposure-time-dependent manner, but the activity of MMP-2 did not change. The results of western blot (Fig. 6b) showed that NTP treatment also significantly decreased the protein expression level of MMP-9, but not MMP-2, in a time-dependent manner. These results indicated that NTP inhibited the proteolytic activity and protein expression of MMP-9.

### NTP inhibited phosphorylation of ERK1/2 and JNK in HeLa cells

MAPKs, including ERK1/2, p38 and JNK, regulate cell invasion as well as migration in various cell types^23^,^29^,^30^. To elucidate the mechanisms responsible for the inhibitory effect of NTP on metastasis, phosphorylation of MAPKs in HeLa cells was measured by western blot. The results (Fig. 7) showed that NTP exposures significantly decreased the phosphorylation of ERK1/2 and JNK in an exposure-time-dependent manner but not the total level of these two proteins, whereas no distinct change was observed in the phosphorylation level of p38. These results suggested that NTP inhibited the metastatic activity of HeLa cells *via* inactivating JNK and ERK1/2 signaling pathways.

### NTP inhibits HeLa cells invasion by suppressing phosphorylation of JNK and ERK1/2

We proceed to further confirm whether the NTP-induced changes of MAPK signaling pathway were directly related to NTP-dependent HeLa cell invasion. The cells were pretreated with JNK inhibitors (SP600125), ERK1/2 inhibitors (SCH772984) or p38 MAPK inhibitors (SB203580) for 2 h and then exposed to NTP for 10, 20 or 40 s. As shown in Fig. 8, treatment with NTP alone or MAPK inhibitors significantly suppressed HeLa cell migration, as compared with that of the control. Furthermore, NTP synergistically suppressed migration after pre-treating with ERK1/2 and JNK inhibitors, but not so with the p38 MAPK inhibitor. The result illustrated that ERK1/2and JNK signaling pathways played a key role in HeLa cell migration.

### Expression of MMP-9 was partly dependent on ERK1/2 and JNK activities in HeLa cells

To determine the role of MAPK signaling pathway in MMP-9 expression of HeLa cells, we evaluated MMP-9 expression in HeLa cells using MAPK inhibitor supplementation. Western blot results (Fig. 9) showed that inhibitors of p38MAPK, ERK1/2 and JNK all reduced MMP-9 expression. In addition, NTP could synergistically down-regulate MMP-9 expression with the ERK1/2 inhibitor and the JNK inhibitor, but not with the p38MAPK inhibitor. The results suggested that inhibition of MMP-9 expression by NTP could be mediated through inactivation of ERK1/2 and JNK signaling pathways in HeLa cells.

## Discussion

NTP has been extensively studied for its biomedical applications and has recently emerged as a potential novel tool in cancer treatment. Previous studies focused mainly on the apoptotic cancer cell death mediated by NTP as a potential cancer therapy strategy^5^. However, the mechanisms involved in the NTP-induced inhibition of cell migration and invasion have not been elucidated. In the present study, we investigated the inhibitory effects of NTP on the migration and invasion of human cervical cancer HeLa cells, and the underlying mechanisms involved in this process. Our results provided evidence that NTP exerted an anti-tumor effect *via* inhibiting cancer cell migration and invasion.

Invasion and migration are important features of malignant tumors^18^. Tumor metastasis remains the main cause of treatment failure and death in a variety of tumors. To identify the anti-metastatic effects of NTP, we compared the migratory and invasive activity of HeLa cells using the scratch wound healing, transwell migration assay, and matrigel invasion assay. Our results showed that NTP significantly inhibited the migration and invasion of HeLa cells. These results were consistent with previous findings that NTP treatment decreased cell migration and invasion in several cell types.

MMPs, a family of zinc-binding proteases, can degrade the extracellular matrix (ECM) and basement membrane for cancer cells to enable migration and invasion^27^,^28^. Among MMPs, expressions of MMP-2 and MMP-9 are high in various malignant tumors and are closely related to tumor migration^28^. Therefore, early suppression of expression and/or proteolytic activity of MMP-9/2 can be the target for preventing cancer metastasis. To further explore the specific effects of NTP on MMP-2 and MMP-9, Gelatin zymography assay was used to detect the activities of MMP-2 and MMP-9 in HeLa cells. The results showed that NTP inhibited activities of MMP-9 in a time-dependent manner. The results of western bolt further revealed that the reduction of MMP-9 activity was a result of down-regulation at the protein level. These results suggested that NTP could inhibit or delay cancer invasion and migration in HeLa cells *via* reducing MMP-9 expression and activity.

Previous reports from various laboratories demonstrated that MMP-9 expression was critically mediated by the MAPK pathway in various cell lines^23^,^31^. The activation of ERK1/2 and/or p38 MAPK played important roles in controlling MMP-9 gene expression through stimulating transcription factors (AP-1 and NF-κB)^24^,^30^. The JNK signaling was essential for a variety of biological processes such as morphogenesis, cell proliferation, migration, invasion and cell death^32^,^33^. Several studies indicated that suppression of MAPKs had the potential to prevent invasion and metastasis for various tumors^23^,^24^. Our results showed that NTP exposures inhibited phosphorylation of ERK1/2 and JNK in a time-dependent manner. These results suggested that NTP inhibited the metastatic activity of HeLa cells *via* inactivating the MAPK pathway. However, how NTP inhibited these intracellular signal pathways to initiate the response remained unclear to date. Previous studies also demonstrated that reactive oxygen species (ROS) generated by NTP had selective damages on cancer cells through induction of apoptosis or loss of cell adhesion^7^,^34^,^35^. Extracellular ROS could activate cell surface receptors to regulate cell migration and invasion^36^,^37^. Various chemical or physical stimulators could regulate MMP-9 expression *via* increasing the ROS level^29^,^36^. Based on the above discussion, it was postulated that ROS generated by NTP could be the most effective major factors to initiate the suppressive effect of NTP on cell migration and invasion. Nevertheless, further studies to investigate the signaling initiated by NTP would be needed for a better understanding on the mechanism of NTP inhibition of migration and invasion.

In conclusion, our results demonstrated that NTP exposure effectively inhibited the migration and invasion of human cervical cancer HeLa cells *via* inhibiting the phosphorylation of JNK and ERK1/2, which led to down-regulation of MMP-9 activity and expression. It is anticipated that these results will provide a mechanistic insight into the potential effects of NTP on the suppression of cervical cancer invasion and metastasis.

## Methods

### Cell culture and reagents

Human cervical cancer HeLa cells (ATCC, CCL-2) were obtained from American Type Culture Collection and cultured in DMEM supplied with 10% FCS, 100 U/mL of penicillin and 100 μg/mL of streptomycin. All cultures were maintained in a 37 °C and 5% CO_2_ humidified atmosphere. Matrigel was purchased from BD Biosciences (Bedford, MA). The primary antibodies for ERK1/2, p-ERK1/2, JNK, p-JNK, p38, p-p38, MMP-2, MMP-9, Bax, Bcl-2, Caspase-3, Bid, cytochrome *c* and β-actin were purchased from Cell Signaling Technology Inc. (Beverly, MA, USA). Horseradish peroxidase (HRP)-conjugated secondary antibody was purchased from Santa Cruz Biotechnology (Santa Cruz, CA, USA). FITC-conjugated phalloidin was purchased from Sigma (Sigma -Aldrich, St. Louis, MO). γ-H2AX antibody was purchased from Abcam (Abcam, Cambridge, MA, USA). BCA Protein Assay Kit and enhanced chemiluminescence (ECL) reagents were purchased from Pierce (Rockford, IL, USA). Cell counting kits-8 (CCK-8), Annexin V-FITC/propidium iodine (PI) apoptosis detection kit, JC-1 Mitochondrial Potential Detection Kit, RIPA lysis buffer and phenylmethyl sulfonylfluoride (PMSF) were purchased from Beyotime Inst. Biotech (Beijing, China). DMEM medium was purchased from Invitrogen Life Technologies (Carlsbad, CA, USA). Fetal calf serum (FCS) was purchased from Thermo Scientific (Rockford, IL, USA). Polyvinylidene difluouride (PVDF) membrane were purchased from Millipore Corp (Bedford, MA, USA). MAPK inhibitors (ERK1/2 inhibitor SCH772984, p38 MAPK inhibitor SB203580 and JNK inhibitor SP600125) were purchased from Selleck Chemicals (Houston, TX, USA). All other chemicals and reagents were of the highest quality and obtained from standard commercial sources.

### DBD plasma device

The atmospheric pressure dielectric barrier discharge (DBD) plasma was schematically illustrated previously^25^. The four DBD plasma reactors were sealed in a hollow plexiglass cylinder as a reactor chamber with two air orifices. One was used to inject the working gas, while the other was used to expel air from the hollow plexiglass cylinder. The high voltage electrode was a 32 mm diameter copper cylinder, which was covered by 1 mm thick quartz glass as an insulating dielectric barrier. The ground electrode was a 37 mm diameter copper cylinder. The discharge gap between the bottom of the quartz and the treated sample surface was fixed at 5 mm. The alternating current power supply was a commercial transformer capable of continuous and tunable output voltages and frequencies. The applied voltage and discharge current of the DBD plasma were monitored using a Tektronix MSO 5104 digital oscilloscope equipped with a high voltage probe (Tektronix P6015A) and current probe (Tektronix P6021). Helium gas was injected into the chamber through the gas inlet with a fixed flow rate of 80 L/h. In order to expel as much air as possible from the reactor chamber, helium was injected at 5 min before the experiment. The non-thermal plasma was generated by a voltage of 12 kV (peak to peak) at a frequency of 24 kHz. The discharge power density was measured to be about 0.9 W/cm^2^.

### Non-thermal plasma treatment

For plasma exposures, 3.5 × 10^5^ cells were seeded into 30 mm diameter Petri dishes. The medium was replaced with 2 ml fresh complete culture medium just before exposures. The distance between the nozzle and the surface of culture medium was fixed at 10 mm. The cells were then exposed to NTP for 10, 20 or 40 s. The control cells (NTP exposure for 0 s) were subjected to identical procedures except the plasma treatment. A gas-only treatment (helium) was used to confirm the presence or absence of effects from the gas alone. At the chosen time points, the cells were harvested for further experiments.

### Cell viability assay

The cell viability was measured by using the CCK-8 assay (Beyotime Biotech, China) according to the manufacture’s recommendations. Briefly, HeLa cells (3 × 10^5^ per well) were seeded into 30 mm dishes with 1.8 mL complete culture medium and exposed to NTP for 10, 20 or 40 s. After 24, 48 or 72 h incubation, 200 μL of CCK-8 solution was added into the cell culture medium and incubated for a further 4 h at 37 °C. After plate vibrating for 20 s, the supernatants (100 μL) were transported into a 96-well plate. Absorbance at 450 nm was read with a microplate reader (ELx800, BioTek Instruments Inc., USA).

### Immunocytochemistry

HeLa cells (3 × 10^5^ per well) were seeded into 30 mm dishes with 1.8 mL complete culture medium and exposed to NTP for 10, 20 or 40 s. After 24 h incubation, the cells were fixed with 4% formaldehyde for 30 min. and then permeabilized with 0.1% Triton X-100. After blocking in bovine serum albumin (BSA) in 5% PBS for 45 min, the dishes were incubated with a polyclonal rabbit anti-γ-H2AX antibody (1:50) for 2 h. The dishes were then washed again in PBS and incubated with FITC-labeled goat anti-rabbit antibody (1:200) for 60 min. After rinsing in PBS, DAPI was added to dishes for 10 min to counter stain nuclei. The dishes were washed with PBS and then visualized using a fluorescence microscope (Leica DMI 40008, Germany).

In addition, cytoskeleton staining was performed using FITC-conjugated phalloidin according to the manufacturer’s instructions.

### Mitochondrial transmembrane potential (Δψm) assessment

The mitochondrial transmembrane potential Δψm was analyzed using a JC-1 Mitochondrial Potential Detection Kit (Biotium Inc., Hayward, CA, US). Briefly, HeLa cells (3 × 10^5^ per well) were seeded into 30 mm dishes with 1.8 mL complete culture medium and exposed to NTP for 10, 20 or 40 s. After 24 h incubation, cells were harvested and stained by JC-1 in PBS for 30 min at room temperature in the dark, followed by flow cytometric analysis.

### Flow cytometry analysis of apoptosis

Annexin V-Fluorescein isothiocyanate/PI apoptosis detection kit (KeyGen Biotech Co., Ltd., Nanjing, China) was used for apoptosis detection. Briefly, HeLa cells (3 × 10^5^ per well) were seeded into 30 mm dishes with 1.8 mL complete culture medium and exposed to NTP for 10, 20 or 40 s. After 24 h incubation, cells were collected and washed twice with PBS, and then suspended with 500 μL of 1× Annexin V binding buffer containing 5 μL of Annexin V-FITC and 5 μL of PI. After incubation in the dark for 10 min at room temperature, the cells were analyzed using flow cytometry (Beckman Coulter, Fullerton, CA).

### Wound-healing assay

HeLa cells were seeded into 30-mm dishes and grown to 90% confluence. A linear wound was created in the confluent monolayer by using a 200 μL micropipette tip, and followed by washing with PBS to remove the cell debris. The cells with 2 ml culture medium were then exposed to NTP for 10, 20 or 40 s. After 24 h incubation, cell migration was observed under a microscope (Olympus IX71, Tokyo, Japan) at a magnification of 100× . The cells migrated across the black lines were counted in five randomly chosen fields of view in each sample. The inhibition effect was expressed after normalization (taking the amount for the control group as 100%).

### Cell migration and invasion assays

The transwell insert for 24-well plate (8 μm-pore size, Corning, New York, USA) was used to measure the migratory and invasive ability of cells. For transwell migration assays, HeLa cells (2.5 × 10^4^) were seeded into the transwell insert (upper chamber) with serum-free medium after NTP exposure for 10, 20 or 40 s, and the culture medium with 10% FCS was added in the lower chamber (the space between the well bottom and the insert) for chemo-attractant. The invasion assays were performed similarly except that the upper chambers of 24-well cell culture inserts were coated with 200 mg/ml of Matrigel (BD Biosciences, Bedford, MA). After 24 h incubation, the insert was taken out and the cells were fixed with 4% paraformaldehyde for 30 min and stained with 1% crystal violet. The non-invading cells were carefully removed from the upper surface of the insert membrane with cotton wool. The number of cells migrated to the lower surface of the membrane was determined by counting 10 randomly selected fields of view under the microscope. Data were expressed as the percentage of invasion of treated cells as compared to the control cells.

### Gelatin zymography

Gelatin zymography was performed with the MMP Zymography assay kit (Applygen Technologies Inc.) to measure the activities of MMP-9 and MMP-2 according to the manufacturer’s instructions. Briefly, HeLa cells were washed with PBS, and then serum-free culture medium was added before the NTP exposure for 10, 20 or 40 s. After 24 h incubation, the supernatants were electrophoresed on 8% SDS-PAGE gels containing 0.1% gelatin. The gels were washed twice with washing buffer (2.5% Triton X-100) for 1 h to remove SDS, and were then incubated in developing buffer (50 mM Tris-Cl, pH 7.6, 200 mM NaCl, 10 mM CaCl_2_) at 37 °C for 12 h for digestion of gelatin. The gelatinolytic activity of MMP-9 and MMP-2 was visualized by staining the gels with Coomassie blue for 30 min and destaining with 45% methanol/10% acetic acid until clear bands suggestive of gelatin digestion appeared. The subsequent zymographic band intensities were quantified using the QuantityOne software (Bio-Rad, Hercules, CA).

### Western blot analysis

HeLa cells (3 × 10^5^ per well) were seeded into 30-mm dishes with 2 mL complete culture medium and then exposed to NTP for 0, 10, 20 and 40 s. After 24 h incubation, the total protein was extracted from NTP-treated cells as described previously^38^. The protein concentration was determined with the BCA Protein Assay Kit (Pierce, Rockford, IL, USA). Equivalent amounts of protein samples were uploaded and separated by 12% SDS-PAGE, and then electro-transferred to polyvinylidene difluouride (PVDF) membrane (Millipore Corp, Atlanta, GA, US). The membranes were blocked in 5% non-fat dry milk at room temperature for 1 h, and then incubated with primary antibodies overnight at 4 °C, followed by HRP-conjugated secondary antibodies at room temperature for 1 h. The signals were developed using the ECL (enhanced chemiluminescence) reagents (Pierce, Rockford, IL, USA) and exposed to an X-ray film (Kodak, Tokyo, Japan). Each band was quantified by densitometric scanning using the free software ImageJ. The densitometry readings of the bands were normalized to β-actin expression.

### Statistical analysis

All data were expressed as mean ± standard deviation (S.D). The difference between the treated samples and the untreated controls was analyzed by Student’s *t*-test and those differences corresponding to *p* < 0.05 were considered significant.

## Additional Information

**How to cite this article**: Li, W. *et al.* Non-thermal plasma inhibits human cervical cancer HeLa cells invasiveness by suppressing the MAPK pathway anddecreasing matrix metalloproteinase-9 expression. *Sci. Rep.* **6**, 19720; doi: 10.1038/srep19720 (2016).

## Figures and Tables

**Figure 1:** Effects of NTP on the growth of HeLa cells. HeLa cells were exposed to NTP for 10, 20 or 40 s. Data are expressed as means ± S.D. for three independent experiments with triplicate each. *p < 0.05; **p < 0.01 versus control (NTP exposure time for 0 s).

**Figure 2:** Effects of NTP on DNA damage, apoptosis, mitochondrial transmembrane potential (Δψm) and cytoskeleton in HeLa cells. (**a**) Immunocytochemistry of γ-H2AX in cells and number of γ-H2AX foci per cell at 24 h after NTP treatment. DAPI was used to stain the cell nuclei. Scale bar = 20 μm. (**b**) Annexin V-FITC/PI staining assay was used to determine the percentage of apoptotic cells in NTP-treated Hela cells. (**c**) The Δψm was analyzed using a JC-1 Mitochondrial Potential Detection. (**d**) Immunofluorescence assays using FITC-conjugated phalloidin were performed to visualize the cytoskeleton (F-actin), and DAPI was used to stain the cell nuclei. Each data point represents the mean ± S.D. from three independent experiments. Scale bar = 20 μm. *p < 0.05; **p < 0.01 versus control (NTP exposure time for 0 s).

**Figure 3:** Effects of NTP on the expressions of Bax, Bcl-2, Caspase-3, Bid, cytochrome c and γ-H2AX in HeLa cells. The cells were exposed to NTP for 10, 20 or 40 s. After 24 h incubation, total protein was extracted and subjected to SDS-PAGE, followed by western blot analysis. The internal control was β-actin.

**Figure 4:** Effects of NTP on migration of HeLa cells. All cell images were captured with 100× magnification. The relative migration of each sample was calculated from the difference in the area of unclosed wound region measured as compared to those of the untreated control (NTP exposure time for 0 s). Data are expressed as means ± S.D. for three independent experiments with triplicate each. *p < 0.05; **p < 0.01 versus control (NTP exposure time for 0 s).

**Figure 5:** Effects of NTP on invasion and migration of HeLa cells. All the cell images were captured with 100× magnification. Data are expressed as means ± S.D. for three independent experiments with triplicate each. *p < 0.05; **p < 0.01 versus control (NTP exposure time for 0 s).

**Figure 6:** Effects of NTP on the proteolytic activities and protein expression levels of MMP-9 and MMP-2 in HeLa cells. (**a**) The activities of MMP-9 and MMP-2 were measured by gelatin zymography. Densitometric analysis of the clear bands on the zymograms was performed using the Quantityone software. (**b**) The expressions of MMP-9 and MMP-2 were detected by Western blot analysis and quantified using the ImageJ program. The densitometry readings of the bands were normalized to β-actin expression. Each data point represents the mean ± S.D. from three independent experiments. *p < 0.05; **p < 0.01 versus control (NTP exposure time for 0 s).

**Figure 7:** Effects of NTP on the MAPK pathway in HeLa cells. The cells were exposed to NTP for 10, 20 or 40 s. After 24 h incubation, total protein was extracted and subjected to SDS-PAGE, followed by Western blot analysis. β-actin was used as an internal control. The expressions of ERK1/2 and p-ERK1/2 (**a**), JNK and p-JNK (**b**), p38 MAPK and p-p38 MAPK (**c**) proteins were determined using Western blot analysis and quantified using the ImageJ program. The upper panel shows a representative Western blot result. The lower panel illustrated the fold difference of integrated absorbance of protein after normalization with β-actin. Each data point represents the mean ± S.D. from three independent experiments. *p < 0.05; **p < 0.01 versus control (NTP exposure time for 0 s).

**Figure 8:** Effects of NTP and MAPK inhibitors on migration of HeLa cells. The cells were pretreated with or without MAPK inhibitors (ERK1/2 inhibitor SCH772984, p38 MAPK inhibitor SB203580 and JNK inhibitor SP600125) for 2 h. The cells were then exposed to NTP for 20 s. After 24 h incubation, the migration of HeLa cells with different treatments was tested by cell migration assay. The data represent the mean ± S.D of three independent experiments. *p < 0.05, **p < 0.01.

**Figure 9:** Effects of NTP and MAPK inhibitors on MMP-9 expression of HeLa cells. The cells were pretreated with or without MAPK inhibitors (ERK1/2 inhibitor SCH772984, p38 MAPK inhibitor SB203580 and JNK inhibitor SP600125) for 2 h. The cells were then exposed to NTP for 20 s. After 24 h incubation, the protein levels of MMP-9 were determined by Western blot. The data represent the means ± S.D. of three independent experiments. The lower panel illustrated the fold difference of integrated absorbance of protein after normalization with β-actin. *p < 0.05; **p < 0.01.
